# Risk Factors of Composite Attachment Loss in Orthodontic Patients during Orthodontic Clear Aligner Therapy: A Prospective Study

**DOI:** 10.1155/2021/6620377

**Published:** 2021-01-23

**Authors:** Chen Yaosen, A. M. Mohamed, Wang Jinbo, Zheng Ziwei, Maher Al-balaa, Yang Yan

**Affiliations:** ^1^MDS Orthodontic Section of Stomatology Department, Zhongnan Hospital, Wuhan University, Wuhan, China 430000; ^2^Master of Nursing Department, Zhongnan Hospital, Wuhan University, Wuhan, China 430000; ^3^College of Stomatology, Hubei University of Science and Technology, Xianning, China 437000; ^4^MDS Orthodontic Section of School of Stomatology, Wuhan University, Wuhan, China 430000; ^5^Stomatology Department, Zhongnan Hospital, Wuhan University, Wuhan, Hubei 430000, China

## Abstract

**Background:**

The composite attachment loss during orthodontic clear aligner therapy is an adverse event that commonly happens in our daily practice. However, there is a lack of related statistical analysis and studies analyzing the related risk factors. Therefore, the aim of this study is to assess the incidence of attachment loss during orthodontic clear aligner therapy and to identify rick factors that may predict such event.

**Materials and Methods:**

The demographics and clinical variables of 94 patients undergoing clear aligner therapy (27 males and 67 females; average age: 27.60 ± 0.86 years) were recorded. Both patient-related and tooth-related attachment loss was recorded. The chi-squared test and logistic regressive analysis were applied to identify the potential risk factors. SPSS for Mac (version 23.0, IBM, USA) was used for statistical analyses. *P* < 0.05 was considered statistically significant.

**Results:**

Our study suggested that the risk factors for attachment loss include frequent aligner removal (≥ 5 times a day) (losing rate = 60.0%, *P* = 0.005), aligner wear time less than 18 hours a day (losing rate = 50.8%, *P* = 0.014), eating without aligners inserted (losing rate = 47.9%, *P* = 0.034), utilizing aligner tray seaters (losing rate = 48.2%, *P* = 0.006), and unilateral mastication (losing rate = 52.1%, *P* = 0.002). The multivariable logistic regression analysis indicates that aligner wear time less than 18 hours a day (*P* = 0.020, *B* = 0.925), using aligner tray seaters (*P* = 0.007, *B* = 1.168), and unilateral mastication (*P* = 0.034, *B* = −0.458) were considered independent factors that can predict the composite attachment loss in orthodontic clear aligner therapy.

**Conclusion:**

Wearing aligner less than 18 hours a day, using aligner tray seaters, and unilateral mastication may contribute to increased incidence of composite attachment loss during orthodontic clear aligner therapy.

## 1. Background

Clear aligner orthodontic treatment is a quickly growing sector in orthodontic technology due to the increasing demand [1, 2]. Since Align Technology Inc. first introduced the Invisalign to the orthodontic market, as one of the pioneers of clear aligner therapy, many different types of clear aligners have been developed and became commercially available. With the help of these devices, orthodontists are able to treat a wide range of malocclusions, from mild crowding to more severe cases [3].

Although orthodontic fixed appliances have become smaller and more esthetically acceptable over the years, they still receive more critics than clear aligner for their unpleasant look and the inconvenience of using. In addition, studies have found clear aligners may be more amenable to periodontal health than fixed appliances; thus, they are recommended for patients at high risk of developing gingivitis [4, 5]. Besides, Guo et al. found that clear aligners can induce nonpathogenic changes of the subgingival microbiome in the first three months of treatment [6]. Furthermore, it has been reported that patients treated with aligners may experience less root resorption and less risk of developing white spot lesions (WSLs) comparing to traditional fixed appliances [7, 8].

The clear aligner therapy differs from traditional fixed appliances in that clear aligners rely on a series of appliances fabricated from a transparent polymer that covers the teeth. The dentition is planned for movement with a computer-aided design to prescribe varying amounts of corrections to the individual teeth [9].

Aligner attachments serve as an important auxiliary device for many clear aligners to transfer the forces from the aligner to the tooth root and crown. In most cases, attachments are automatically placed in specific locations on teeth that determined by the computer algorithm, and they control the application point of the force, the direction of the force, and the amount of force applied. Aligner attachments have different shapes that help to increase the retention and provide better control of certain tooth movements whenever needed [10]. Attachments consist of composite resin bonded to the tooth surface. Bond failure or patient neglect can cause attachment loss from the tooth surface. Attachment loss can induce significant clinical problem that may prolong treatment time, increase the number of revisit, and the prognosis of the treatment [11].

There are risk factors, including operator-related and patient-related factors, that may result in attachment loss. A recent study demonstrated that the traditional attachment and frequent aligner removal (more than or equal to five times a day) may lead to attachment loss. On the other hand, wearing aligners while eating may prevent attachment loss [12]. There are many studies available investigating the effects of clear aligner orthodontic treatment, but the incidence of composite attachment loss and its influence in clear aligner therapy has not been well studies. Therefore, the aim of the present study is to assess the incidence of composite attachment loss and analyze its risk factors in clear aligner orthodontic treatment.

## 2. Materials and Methods

The protocol of this prospective investigation was granted by the Institutional Review Board at Zhongnan Hospital of Wuhan University (code number 2019054). All methods were performed in accordance with the relevant guidelines and regulations or Declaration of Helsinki as patients were involved. Written informed consent was obtained from all subjects or, if subjects are under 18, from a parent and/or legal guardian. Patients of the orthodontic department in Zhongnan Hospital of Wuhan University were screened. Inclusion criteria were (1) started treatment from 2017.9 to 2018.12; (2) received comprehensive clear aligner (Invisalign, Align Technology, USA) treatment of upper and lower arches; (3) no previous orthodontic treatment; (4) no dental fluorosis, enamel hypoplasia, dentin hypoplasia, or other abnormal teeth structure; (5) no bruxism; (6) no full coverage crowns or buccal restorations; and (7) no occlusal or attachment interference in initial occlusion. A total of 94 patients (27 males and 67 females; average age: 27.60 ± 0.86 years) were enrolled in this investigation.

### 2.1. Bonding Method

Before delivery of the first aligner, each patient was given a set of passive thermoformed retainers with proper instruction. After two weeks, the template appliance was used to make bond attachments.

Before bonding, the template appliance was wiped with 75% ethyl alcohol and air-dried. After that, the patients' teeth were polished using a fluoride-free prophylaxis paste on a rubber cup attached to a low-speed handpiece. The buccal enamel surfaces of the teeth were etched with 35% orthophosphoric acid (Gluma, Heraeus Kulzer GmbH, Germany) for 30 seconds, rinsed with water for 30 seconds, and dried with an air stream to ensure complete removal of the etchant. The bonding agent (Adper SingleBond2, 3M ESPE, USA) was then applied to the buccal surface and light cured for 10 seconds using a Woodpecker light-curing unit (1000-1200 mW/cm^2^; Foshan, Guangdong, China). Then, composite resin (Filtek Z350XT, 3M ESPE, USA) was applied to the attachment wells of the clear aligner template appliance. The template was pressed on the tooth surface and light cured for 40 seconds using the same light-curing unit. Extra composite resin was removed with a high-speed handpiece and finishing bur. All the procedures were carried out by the same experienced doctor and his assistant according to the manufacturers' instructions. All the patients received standardized oral hygiene education, including the recommendation to brush their teeth before sleeping and after eating. Patients were asked to record the removal frequency and daily wear time at least 14 days after the bonding.

### 2.2. Data Collection

After bonding, the patients were instructed to inform and visit the clinic immediately in case of attachment loss or breakage. Electronic questionnaire's link was sent to each patient by email at the beginning of the treatment. The outcome would be delivered to researchers automatically once the questionnaire was completed. At revisit, the following information was confirmed and gathered by researchers: (1) tray progression before the attachment loss, (2) the position of the attachment that was lost (verified by the doctor), (3) the causes of the attachment loss, (4) the average daily aligner removal frequency, (5) the average daily wear time, (6) masticatory habits, (7) eating habits, (8) the method of appliance removal, (9) use of any aligner tray seaters, and (10) eating with or without the clear aligners.

### 2.3. Statistical Analysis

Both patient-related and tooth-related incidences of attachment loss rates were calculated. The chi-squared test was used to compare the categorical variables. The intraclass correlation coefficient generated by kappa statistics was adopted to assess the agreement between two measurements. The logistic regressive analysis was applied to identify the risk factors for attachment loss. Statistical analyses were performed using the SPSS software for Mac (version 23.0, IBM, USA), with *P* values of less than 0.05 considered as statistically significant.

## 3. Results

During the study, 54 patients experienced at least one attachment loss were included, and a total of 94 attachments loss were recorded. The overall incidence of patient-related attachment loss was 57.45% while the incidence of tooth-related attachment loss was 6.74%. A total of 1397 attachments were applied, and the mean number of attachments per patient was 14 ± 0.96. No significant difference was observed between patients experienced attachment loss and those who did not in age, gender, location of the attachments (maxillary or mandibular, left or right), and number of attachments (*P* > 0.05). The attachment characteristics and clinical variables of the patients are summarized in Table 1.

There were 94 attachments lost during the study, including 34 incisor/canine attachments, 20 premolar attachments, and 40 molar attachments, representing 36.1%, 21.3%, and 42.6% of the total attachments lost, respectively. We observed a significant difference of attachment loss rates between attachments at different locations. Specifically, the attachment loss rate in incisor/canine attachments was 7.54%; the rate in premolar attachments was 3.34% and the rate in molar attachments at 11.49%.

The incidence of attachment loss and its potential contributing patient-related factors are summarized in Table 2. Correlations between these variables and attachment loss rate were analyzed using univariate analyses (Table 2) and multivariable logistic regression (Table 3).

Table 2 shows the result of *χ*^2^ analyses/univariate analyses. There are 6 potential factors that affect the rate of attachment loss, including attachment amount, eating with aligners inserted, time of wear, frequency of aligner removal, use of aligner tray seaters, and masticatory habits.

Table 3 summarizes the results of logistical regressive analysis. Aligner wear time (*P* = 0.020, *B* = 0.925), use of aligner tray seaters (*P* = 0.007, *B* = 1.168), and masticatory habits (*P* = 0.034, *B* = −0.485) prominently affected attachment loss in clear aligner orthodontic treatment. Removal frequency (*P* = 0.057, *B* = −0.848) and eating with aligners (*P* = 0.333, *B* = −0.398) did not reach significance in the test.

## 4. Discussion

Clear aligner attachment helps to increase the retention of the trays thus provide better control over tooth movements. Attachment loss during treatment may compromise such benefit and increase the need for refinement [13]. In this study, we identified several risk factors that may affect attachment loss rate. In summary, they can be separated into 3 groups:

1. *Clinical Variables*. Age, gender, the number of attachments, the location of attachment (maxillary or mandibular, left or right, incisor/canine, premolar or molar), and the shape of attachment.
2. *Operator-Related Variables*. Bonding protocol and bonding materials. Once bonding failure occurs, the attachment will detach from the tooth in a short time [14].
3. *Patient-Related Variables*. Aligner removal frequency and method, aligner wear time, use of aligner tray seaters, having food with aligners, and masticatory habits.

In general, the patient-related causes of attachment loss, including aligner removal frequency and method, aligner wear time, use of aligner tray seaters, having food with aligners, and masticatory habits, accounted for 56.25% of total attachment loss. On the other hand, the tooth-related reasons that result in attachment loss were 6.73%, which is lower than the finding of Huang et al. [12] at 16.41%.

### 4.1. Position

Our findings suggest the different locations of attachment, whether maxillary or mandibular, left or right, did not affect the attachment loss rate. However, the attachment loss rate may be influenced by different tooth positions (anterior, premolar, and molar were 7.54%, 3.34%, and 11.49%, respectively). The highest rate of loss occurs with molar attachments, which may due to its special shape that is unfit for bonding attachments, in which the position of the height of contour of the buccal surface is far from the cervical [15, 16]. Such unique position of the molar increases the impacting forces delivered to the attachment in the process of wearing and removing the clear aligners. On the other hand, the operating space when performing molar attachment is limited, and it is difficult to keep the buccal surface isolated during bonding.

### 4.2. Having Food with Aligners Inserted

Our data showed that patients having food with aligners inserted had lower rate of attachment loss. The presence of the clear aligner may buffer the masticatory force on the attachments while eating as well as divert the direct impact of eating hard foods. In addition, the impact force of the food and chewing force of single attachment can be dispersed along the entire dentition, thus greatly reducing the force applied on individual attachment. Therefore, having food with aligner can reduce the probability of attachment loss. However, Moshiri et al. [17] suggest to avoid having food with aligners inserted to prevent white spot lesions (WSLs) during aligner therapy. The manufacturers of clear aligners also advise patients to remove aligners before eating, for both hygiene purposes and to protect the clear aligner material against food with high temperature which may reduce the lifetime of aligner. Other groups have shown that the softness of food did not directly affect the probability of attachment loss [18–20]. Future studies consist of larger population are needed to further investigate the influence of food intake on aligner therapy.

### 4.3. Using Aligner Tray Seaters

Aligner tray seaters, or Chewies, are a type of special appliance comprised of dense foam or plastic designed for clear aligner orthodontic treatment. The use of aligner tray seaters can make the aligners fit more closely with the tooth surface and achieve the intended orthodontic force system [21]. At the same time, the masticatory muscles are exercised with aligner tray seaters for patients who have had extracted premolars or molars, and the unjoyful appearance of “bracket face” can also be ameliorated [22]. However, our finding shows that the use of aligner tray seaters will increase the probability of attachment loss, which is in contrast with the findings of Huang et al. [12]. Even though the clear aligners fit more closely with the attachment after using tray seaters, it may result in an occlusal force that being focused on a single tooth or attachment, which may then increase the attachment loss rate.

### 4.4. Aligner Removal Frequency

Each time the patient inserts or removes the aligner, it will produce an additional dislocation force on the attachments. When the dislocation force is greater than the bonding force, the attachment will separate from the tooth surface. The more frequently the aligner is removed and inserted, the more frequently the attachments are stressed [23, 24]. All 94 lost attachments in this study occurred during removal of the aligners. From the results of the study, the frequency of removing less than 5 times a day did not increase the probability of the attachment loss. However, frequently removal (≥ 5 times a day) is a prominent risk factor of attachment loss.

### 4.5. Wear Time

Clear aligner manufacturers recommend keeping the aligners inserted at least 22 hours a day. However, we found it is difficult to ask our patients meet such requirements on our daily practice. Thus, we studied the influence of wear time on the attachment loss rate. The result showed that wearing the aligners less than 18 hours a day increased the probability of attachment loss. Tooth movement requires sufficient time and suitable forces to achieve desired results [25, 26]. Based on this result, the risk of attachment loss can be reduced by prolonging the duration of aligner wear [27].

### 4.6. Mastication Habit

Bilateral alternate mastication is considered healthy chewing habits under physiological conditions, which has a protective effect on the temporomandibular joint and is also conducive to the balance of occlusal relationship between bilateral posterior teeth [28, 29]. For patients with bilateral alternate mastication, the probability of attachment loss on either side should be similar, which is verified by our data. For patients with unilateral mastication, the occlusal function of the functional side is greater than that of the opposite side. When eating with the appliance inserted, the aligner on the functional side fits more closely with the tooth surface [30], and the difference between the actual tooth movement and the prescription value is smaller. Therefore, the attachment loss rate is also lower than opposite side. The results suggest that unilateral chewing should be avoided, and patients should establish the habit of alternating chewing on both sides.

### 4.7. Limitation of This Research

The data was mostly depending on patients' report, and multiple of these factors likely happened simultaneously without patient's acknowledgement. Therefore, in vitro studies such as finite element analysis need to be used to validate the factors that significantly contributed to attachment loss [31].

## 5. Conclusion

The attachment loss rates of different tooth positions are different which the highest rate occurs with molar attachments and lowest lost rate with premolar attachments. Aligner wear time, chew habits, and use of aligner tray seaters are all influencing factors of attachment loss in clear aligner orthodontic treatment. Our findings suggest that wearing aligners more than 18 hours a day and reducing use of aligner tray seaters may be beneficial for patients undergoing clear aligner orthodontic treatment. Additionally, a unilateral chewing habit may increase the risk of attachment loss. The majority of the risk factors we identified in this study are patient related and can be avoided after a better education.

## Figures and Tables

**Table 1:** Univariate analyses of attachment loss rate (base on attachments).

Factors	No. of attachments	Attachments		Rate (%)	*χ^2^* value	*P* value
		Lost	Retained			
Arch					0.032	0.915
Maxillary	740	50	690	6.76		
Mandibular	657	44	613	6.70		
Side					0.006	1.000
Left	704	47	657	6.68		
Right	693	47	646	6.78		
Tooth position					24.472	0.0001
Incisor/canine	451	34	417	7.54		
Premolar	598	20	578	3.34		
Molar	348	40	308	11.49		

**Table 2:** Univariate analysis of influencing factors of attachment loss.

Factors	No. of cases (attachments)	Attachments		Rate (%)	*χ^2^* value	*P* value
		Lost	Retained			
Gender					0.432	0.566
Male	27 (366)	14 (25)	13 (341)	51.9 (6.8)		
Female	67 (1031)	40 (69)	47 (962)	59.7 (6.7)		
Attachment amount					0.009	1.000
≤ 15	50 (631)	28 (51)	22 (580)	56.0 (8.1)		
>15	44 (766)	26 (43)	18 (723)	59.1 (5.6)		
Eat with aligners					5.029	0.034
Yes	40 (601)	18 (28)	22 (576)	45.0 (4.7)		
No	54 (796)	36 (66)	18 (760)	66.7 (8.3)		
Time per day					6.237	0.014
<18 hours	46 (668)	32 (58)	14 (610)	69.6 (8.7)		
≥ 18 hours	48 (729)	22 (36)	26 (693)	45.8 (4.9)		
Removal frequency					8.524	0.005
<5 times	66 (1020)	32 (65)	34 (955)	48.5 (6.4)		
≥ 5 times	28 (377)	22 (29)	6 (348)	78.6 (7.7)		
Aligner tray seaters					7.754	0.006
Yes	63 (925)	31 (73)	22 (852)	49.2 (7.9)		
No	31 (472)	13 (21)	18 (451)	41.9 (4.5)		
Removal method					0.015	1.000
From buccal	43 (651)	24 (40)	19 (611)	55.8 (6.1)		
From lingual	51 (746)	30 (54)	21 (692)	58.8 (7.2)		
Masticatory habits					10.376	0.002
Unilateral	54 (818)	37 (58)	28 (760)	68.5 (7.1)		
Bilateral	40 (579)	17 (36)	23 (573)	42.5 (6.2)		

**Table 3:** Multivariable logistic regression analysis of attachment loss (based on patients).

Factors	*B* value	S.E.	Wald	*P* value	Exp (*B*)
Removal frequency	-0.848	0.445	3.631	0.057	0.428
Wear time	0.925	0.397	5.417	0.020	2.521
Aligner tray seaters	1.168	0.433	7.266	0.007	3.216
Eating with aligners	-0.398	0.411	0.938	0.333	0.671
Masticatory habits	-0.485	0.229	4.473	0.034	0.615
Constant	0.082	1.241	0.004	0.948	1.085

## Data Availability

The datasets used and analyzed during the current study are available from the corresponding author on reasonable request.
